# Preliminary Evaluation of Artificial Intelligence-Based Anti-Hepatocellular Carcinoma Molecular Target Study in Hepatocellular Carcinoma Diagnosis Research

This article has been retracted.

**DOI:** 10.1155/2022/8365565

**Published:** 2022-09-19

**Authors:** Yuan Wang, Chao Wei, Xiangui Deng, Shudi Gao, Jing Chen

**Affiliations:** ^1^Infectious Disease Department, Hospital of Chengdu University of Traditional Chinese Medicine, Chengdu, Sichuan 610072, China; ^2^Qijiang Hospital of The First Affiliated Hospital of Chongqing Medical University, Chongqing 401420, China; ^3^Wenlong Hospital of Qijiang, Chongqing 401420, China; ^4^Taiyuan Hospital of Traditional Chinese Medicine, Taiyuan, Shanxi 030000, China

## Abstract

In this paper, in-depth research analysis of anti-hepatocellular carcinoma molecular targets for hepatocellular carcinoma diagnosis was conducted using artificial intelligence. Because BRD4 plays an important role in gene transcription for cell cycle regulation and apoptosis, tumor-targeted therapy by inhibiting the expression or function of BRD4 has received increasing attention in the field of antitumor research. Study subjects in small samples were used as the validation set for validating each diagnostic model constructed based on the training set. The diagnostic effect of each model in the validation set is evaluated by calculating the sensitivity, specificity, and compliance rate, and the model with the best and most stable diagnostic value is selected by combining the results of model construction, validation, and evaluation. The total sample was divided into a training set and test set by using a stratified sampling method in the ratio of 7 : 3. Logistic regression, weighted *k*-nearest neighbor, decision tree, and BP artificial neural network were used in the training set to construct diagnostic models for early-stage liver cancer, respectively, and the optimal parameters of the corresponding models were obtained, and then, the constructed models were validated in the test set. To evaluate the diagnostic efficacy, stability, and generalization ability of the four classification methods more robustly, a 10-fold crossover test was performed for each classification method. BRD4 is an epigenetic regulator that is associated with the upregulation of expression of various oncogenic drivers in tumors. Targeting BRD4 with pharmacological inhibitors has emerged as a novel approach for tumor treatment. However, before we implemented this topic, there were no detailed studies on whether BRD4 could be used for the treatment of HCC, the role of BRD4 in HCC cell proliferation and apoptosis, and the ability of small molecule BRD4 inhibitors to induce apoptosis in hepatocellular carcinoma cells.

## 1. Introduction

For most multicellular organisms, including humans, cells have a strong intrinsic proliferative capacity for normal development and in vivo homeostasis. For example, in the living state, human GI epithelial cells can divide more than once or twice a day [1]. Thus, there is no rate limit to the proliferative capacity of cells, yet advanced regulatory mechanisms have evolved to limit this excess proliferative capacity to the right time and place, and it is this excess proliferative capacity that lays the foundation for cancer cell formation. With the development of modern medicine, there has been great progress in the diagnosis and treatment of HCC. Surgical resection as well as liver transplantation are radical treatments and remain important options for the treatment of liver cancer. However, due to the insidious onset of hepatocellular carcinoma, early symptoms are not obvious, and about 20% of patients can receive radical resection surgery when they have obvious symptoms, resulting in a poor prognosis. With the introduction of molecularly targeted drugs, the advancement of surgery and the formation of a comprehensive treatment system mainly based on surgery, the treatment of HCC has made a breakthrough, and the five-year survival rate and postoperative quality of life of patients have been greatly improved [2]. The introduction of molecularly targeted drugs, which are more specific to tumor cells and have no or less damage to normal tissues, has not only brought about a fundamental change in the pattern of tumor development but also a fundamental development, with more than 30 types of targeted drugs currently on the market. Cancer cells are mutated cells that cause cancer. Different from normal cells, cancer cells have three characteristics of infinite proliferation, transformation, and easy transfer. They can proliferate indefinitely and destroy normal cells and tissues. In addition to uncontrolled division (which can divide indefinitely), cancer cells also locally invade surrounding normal tissues and even metastasize to other parts of the body via the circulatory system or lymphatic system in the body. If the tumor is small, the disease has not spread beyond the liver, and suitable donor liver tissue can be found, liver transplantation may be an option. Donated liver tissue comes from deceased or living donors. In the case of a living donor, the donated tissue is a portion of the liver, not the entire liver.

Medical imaging artificial intelligence technology is developing rapidly and has become an extremely dynamic new research area. New technologies, represented by image comics and deep learning, have expanded the ability to assist in liver medical imaging beyond the scope of traditional image analysis. Imaging omics, by extracting many high-dimensional image features related to diagnostic results, constructs highly robust prognostic prediction models to screen out potential groups of people with high and low risk of postoperative recurrence, to assist physicians in assessing the near-term efficacy and long-term prognosis of liver cancer against various treatment modalities and precisely formulate individualized treatment plans [3]. Deep learning, as an automatic image analysis method, is often applied to segmentation and volume measurement of liver and liver tumors, tumor detection and tumor classification, and assisting in planning surgery. Imaging omics and deep learning have great potential applications in predicting the prognosis of liver cancer. Hepatocellular carcinoma has a wide range of biological variability, including from very low metastatic potential to highly aggressive phenotypes. Some unique molecular or pathological subtypes of HCC are strongly associated with good or poor prognosis [4]. The classification criteria for hepatocellular carcinoma advocated by pathologists are evolving, and pathology itself is somewhat divergent in terms of histologic grading and assessment of vascular invasion. For hepatocellular carcinoma with atypical imaging manifestations before ablative treatment, puncture biopsy can clarify the nature of the lesion, refine the molecular typing of hepatocellular carcinoma, and provide valuable information for selecting treatment modality and judging prognosis [5]. However, there may be great differences between biopsy results and postoperative pathological results, and the reliability is insufficient. Therefore, imaging-assisted prediction of HCC subtypes before ablative treatment of hepatocellular carcinoma is very important and challenging.

Molecularly targeted drugs mainly target the key targets of the pathophysiological occurrence and development of malignant tumors for therapeutic intervention, and some molecularly targeted drugs have shown good efficacy in the corresponding tumor treatment. Although molecularly targeted drugs have outstanding curative effect on the tumors they target and have good tolerance and mild toxicity, it is generally believed that they cannot completely replace traditional cytotoxic antitumor drugs for a long time. A more common case is a combination of the two. Given the association of steatohepatitis HCC with nonalcoholic steatohepatitis, the incidence of steatohepatitis HCC will further increase as the number of obese patients increases worldwide [6]. Steatohepatitis-type HCC mostly occurs in the context of steatohepatitis and may occur in the absence of HBV or HCV infection and cirrhosis. On imaging, steatohepatitis-type HCC is rich in intratumoral fat and shows diffuse or focal loss of signal intensity on MR inverse phase images. The study of its imaging manifestations is still an area of great interest. There are many deep learning frameworks, such as autoencoders, deep belief networks, and convolutional neural networks. Among them, CNN is the most commonly used in cancer detection, followed by AE and DBN. They are either used to analyze medical images, such as X-rays and CT images, or to analyze molecular-level data, such as gene mutations and gene expression data. At present, deep learning technology cannot be applied to all types of cancers, so existing research generally uses common cancers such as lung cancer and breast cancer as detection targets.

Nanoparticles can be selectively or non-specifically phagocytosed and internalized by cells and distributed in intracellular regions, thus emitting fluorescence in response to specific excitation light for cellular imaging. By exploiting the different affinity properties of molecules and cleverly designing and modifying the structures of discovered molecules, researchers have designed fluorescent materials with the ability to localize to other intracellular sites such as mitochondria, lysosomes, nuclei, cell membranes, and other subcellular structures and detectors with binding effects on specific metal ions and biomolecules. In contrast, AIE fluorescent molecules, which are not limited by the aggregation quenching effect of traditional fluorescent molecules, are more likely to fully demonstrate their photodynamic therapeutic ability for tumors. More importantly, AIE fluorescent molecules are easier to prepare, have stable luminescence performance and good biocompatibility, and are more suitable for clinical application and research than the more studied metal-containing materials such as quantum dots, which have the most basic and indispensable conditions for clinical translation. We believe that AIE nanomaterials are promising to provide better imaging and therapeutic aids for the early diagnosis and treatment of malignant tumors.

## 2. Related Works

There is a need to go beyond current diagnostic forms, recognize the molecular variability driving the biological phenotype, identify imaging features that predict treatment response, and provide a new basis for individualized treatment and thus develop optimal therapeutic strategies [7, 8]. HBP signaling reflects the function of hepatocyte membrane transporters and is regulated by the genetic molecular mechanisms of HCC. The organic transporter for geodetic acid uptake by human hepatocellular carcinoma cells is mainly OATP1B3, located on the basolateral side of hepatocytes. In immunohistochemistry, low uptake of HBP suggests reduced OATP1B3 expression in hepatocytes [9]. Conversely, high HBP uptake suggests that hepatocyte OATP1B3 expression is preserved compared to the hepatic background. The signal intensity of HBP is very sensitive to the extent of hepatocellular carcinoma organic transporter OATP1B3 expression [10]. Wang et al. showed that OATP1B3 expression levels in low-grade heterogeneous nodules were the same as in the surrounding liver, 30% of highly heterogeneous nodules and 75% of early-stage hepatocellular carcinomas had reduced OATP1B3 expression, and all hypo fractionated hepatocellular carcinomas had reduced or absent OATP1B3 expression [11]. However, 6-15% of moderately or highly differentiated hepatocellular carcinomas exhibited high HBP signal due to increased OATP1B3 expression. *β*-strand protein signaling pathway could upregulate OATP1B3 expression in HCC, resulting in significantly higher OATP1B3 expression in some less aggressive hepatocellular carcinomas.

Tipranavir is an inhibitor active against HIV-1 protease and maintains its potency by stabilizing the protease [12]. Tipranavir is a novel non-peptide protease inhibitor with broad antiviral activity against multi-protease inhibitor-resistant HIV-1. In vitro, tipranavir-resistant viruses have a reduced replication capacity that is not ameliorated by the introduction of CA/SP1 cleavage site mutations [6]. In vitro, tipranavir-resistant viruses have a reduced replication capacity that is not improved by the introduction of CA/SP1 cleavage site mutations. In addition to saquinavir, tipranavir-resistant viruses show cross-resistance to other currently approved protease inhibitors [13]. The one-dimensional nanostructures fabricated by printing have unique optical resonance properties in the visible light region. The study found that when the size of one-dimensional nanostructures is larger than the critical value, both scattering and diffraction signals appear in the visible light region, which can significantly amplify the optical signals of nanoscale objects, breaking the traditional optical diffraction limit. Based on the computer-aided drug design amount and its ant hepatocellular carcinogenic activity found in previous tests, our laboratory will investigate its ant hepatocellular carcinogenic activity in depth and lay the foundation for finding new target drugs for the treatment of HCC [14]. Since protein-protein interactions are difficult to be blocked by small molecules, relatively little attention has been paid to proteins bound to histone acetylation markers. This slowly changed with the discovery of the first bromodomain inhibitors. The most effective inhibitors were targeted to the bromodomain and terminal ectodomain families and mimicked the acetyl-lysine fraction, thereby preventing the binding of BET bromodomain proteins to acetylated histones.

Despite their conceptual similarity, imaging omics and deep learning involve completely different technical processes [15]. Imaging omics analysis is based on classical machine learning models in which experts predefine the following: features to be extracted, methods for feature selection, and methods for building classification models. In contrast, deep learning algorithms are based on representational learning and do not use predefined feature engineering. Deep learning algorithms will learn how to remove, process, and combine features to classify the provided training data. Deep learning algorithms based on representational learning have better performance than classical machine learning algorithms when training data is sufficient, but usually require large amounts of training data. Imaging omics and deep learning may extend the complementary capabilities of medical imaging of the liver beyond the scope of traditional visual image analysis. They can obtain additional information about the image that is not available with traditional methods. Imaging histology predicts tumor prognosis by analyzing tumor phenotypes in images. In contrast, deep learning, an automated image analysis method, is often used for organ segmentation and volume measurement, tumor detection, and tumor classification. In recent years, both have shown important applications in the assessment of liver cancer treatment outcomes and prognosis.

## 3. Materials and Methods

### 3.1. Study Subjects and Materials

One group of specimens was preserved in liquid nitrogen immediately after the surgical resection and then frozen at -80°C for protein or RNA extraction; the other group was placed in a specimen lyophilization tube with 4% paraformaldehyde and stored at 4°C then routinely paraffin-embedded and sectioned for histological and pathological analysis. All the above specimens were obtained from patients who had first resected hepatocellular carcinoma, and none of them had received radiotherapy, chemotherapy, or other anti-cancer treatments before surgery [16]. Photoacoustic-fluorescence dual-modality imaging provides highly sensitive real-time visualization for localizing tumors and regional lymph nodes and has outstanding advantages such as non-invasiveness, no ionizing radiation, high spatiotemporal resolution, fast output, and low cost. It can help clinicians accurately locate deep tumors before surgery and quickly determine the extent of lymph node dissection during surgery for precise surgery.

The area where the tissue specimen was located was circled with a marker pen, goat serum blocking solution was added dropwise for 20 min at room temperature, and then diluted primary antibody was added dropwise. After dehydration and transparency, an appropriate amount of neutral gum was added dropwise, and the slides were sealed with coverslips. The images were observed using a light microscope and photographed for preservation, as shown in Table 1.

Cells at the logarithmic growth stage were taken, and cell suspensions were made by conventional digestion and passaged, and counted under the microscope. 5 × 10^5^ hepatocellular carcinoma cells were inoculated in 6-well culture plates and incubated overnight at 37°C and 5% CO_2_ incubator, and after microscopic observation of cell wall attachment the next day, the cells were treated with different concentrations of drugs and placed in the incubator for further incubation. Cells were collected at the time points expected for the assay, and total protein was extracted by lysing cells on ice for 30 min using RIPA lysis solution and centrifuging at 13000 rpm for 20 min [17].

The PVDF membrane was closed with 5% skim milk powder at room temperature for 1 h, then the primary antibody to be tested (1 : 1000 dilution) was added separately, incubated on a shaker at room temperature for 30 min, and then placed in the refrigerator overnight at 4°C. The next day, 1x TBST buffer was used to wash the membrane 3 times, then horseradish peroxidase-labeled secondary antibody working solution (1 : 2000-3000 dilution) was added and incubated on a shaker at room temperature for 1 h. After, 1x TBST buffer was used to wash the membrane fully, the hybridization signal was detected by applying ECL electrochemiluminescence, and the images were saved and analyzed for grayscale values of target protein bands after scanner imaging.

Apoptosis is a kind of programmed death mediated by signaling pathways, which not only exist in the normal physiological state of the body but also play an important role in the development of malignant tumors. The apoptotic signaling pathway in hepatocellular carcinoma cells is severely defective and extremely insensitive to apoptosis induction, which is believed to be one of the most important reasons for the high malignancy of hepatocellular carcinoma and its resistance to conventional radiotherapy.

In this part of the experiment, we investigated the anti-HCC activity of the small molecule BRD4 inhibitor JQ1 and the molecular mechanism of its effect, to elucidate whether inhibition of BRD4 can effectively induce the apoptosis of HCC, as shown in Table 2. Targeted drugs are developed for tumor genes. They can identify characteristic sites on tumor cells determined by tumor cell-specific genes, and by combining with them, block the signal transduction pathways that control cell growth and proliferation in tumor cells, thereby killing tumor cells and preventing their proliferation.

First, this study used the LiTS, a public dataset of liver and hepatocellular carcinoma consisting of data from different clinical sites around the world, which includes portal CT images of 130 patients with HCC or secondary liver tumors, including liver segmentation annotations and liver tumor segmentation annotations. This publicly available dataset was used to train the underlying segmentation model [18]. The preoperative and postoperative CT images of the 63 patients mentioned above were aligned, and the patients who were successfully aligned continued to participate in the study of ablation treatment outcome evaluation. USP has important pathophysiological significance in cardiovascular diseases and can regulate the occurrence and development of important diseases such as atherosclerosis, ischemia-reperfusion injury, familial cardiomyopathy, cardiac hypertrophy, and heart failure. The latest research shows that the important role of UPS is that after it is fully utilized, it can metabolize human waste such as toxins, fat, and cancer cells. In addition, the energy generated by metabolism can stimulate cells to replicate themselves to complete the body's self-metabolic repair. Function.

### 3.2. Diagnostic Analysis of Artificial Intelligence for Liver Cancer

The total amount of contrast agent was 100 ml (Cacique 350 mg/ml, GE Healthcare), and the contrast agent injection rate was 3.5 ml/s. 30 ml of physiological saline was added before and after the injection. The abdominal aortic dynamic monitoring scan was performed with a delay of 15 s and 50 s after reaching the threshold of 150 Hu, respectively [19]. The arterial phase was about 15-25 seconds after injection and the portal phase was about 50-70 seconds after intravenous injection. One CT-enhanced examination was performed before and one after the ablation treatment, and the interval between the two was not more than 14 days.

A total of 252 CT-enhanced images were manually annotated, including pre-and postoperative liver in the arterial and venous phases, preoperative liver tumor, and ablation areas in the postoperative period. When the Dice coefficient was ≥0.8, the segmentation results of H.K were included in the group, and when the Dice coefficient was <0.8, the reviewers H.K and R.R jointly reviewed the images and made reservations until the Dice coefficient was ≥0.8, and the final 3D-R0I outlined by H.K was included in the group. Deep learning algorithms are data-dependent and require large datasets to train. The lack of data in the medical imaging field has created a bottleneck for the application of deep learning in medical image analysis. Medical image acquisition, annotation, and analysis are expensive, and their use is ethically restricted. They also require many resources, such as human resources and funding. This makes it difficult for non-medical researchers to access useful large amounts of medical data.

The network uses residual convolution to improve feature utilization, which not only ensures good performance but also increases the network depth, and the gradient disappearance problem in the deep network is alleviated as the network depth increases [20]. The attention mechanism can be focused on a specific part of the image. By overlaying the attention module, different types of attention can be achieved, thus adaptively changing the features of attention perception. In this study, all the convolutional layers in the liver segmentation network are computed in 2D convolutional form, and a 2D RA-Unit with voxel-level semantic segmentation is constructed and trained; the liver tumor and postoperative ablation area are computed in 3D convolutional form, and a 3D RA-Unit is constructed and trained.

The attention module is used to connect the local features in the encoder and decoder, thus enabling the fusion and reuse of multi-scale features while removing noise. The activation function used in the last layer is an S-type function to generate binary segmentation results, and the rest of the activation functions are linear activation functions, as shown in Table 3.

The liver segmentation results output from the above model were used as the segmentation background to further train the 3D segmentation model of liver cancer lesion and ablation area after treatment. In this study, two 3D RA-Unit models were trained for the segmentation of liver cancer lesions and post-treatment ablation areas, respectively. To overcome the large differences in lesion sizes, 3D patch cascade segmentation networks with dimensions of 20∗30∗30 pixels and 40∗60∗60 pixels were constructed to improve the accuracy of lesion segmentation. Same as the training strategy for the liver, the pre-training of the 3D RA-Unit segmentation model was firstly completed with the publicly available dataset LiTS liver cancer label as the gold standard, and the images used for pre-training were portal phase CT-enhanced images [21]. Finally, a 3D RA-Unet segmentation model of liver cancer lesions and a 3D RA-Unet segmentation model of postoperative ablation area were obtained. In the process of actual development and acquisition of information and data, there will be various reasons for data loss and vacancies. The processing methods for these missing values are mainly based on the distribution characteristics of variables and the importance of variables using different methods. Data cleaning is to achieve the purpose of cleaning by filling missing values, smoothing noisy data, smoothing or removing outliers, and correcting data inconsistencies.

In this study, the safe ablation distance was uniformly set at 5 mm, but the ablation range of tumors located at-risk sites was set to reach the edge of the liver envelope or important blood vessels. Based on the ISD platform, a plug-in for quantitative assessment of the safe ablation boundary was optimized to visualize the ablation effect and measure the required meridians. After successful alignment of pre- and post-ablation CT images, the segmentation results of the liver cancer lesion and the segmentation results of the ablation zone are combined in the same image coordinate system, and the plug-in automatically measures the distance between the axial, coronal, and sagittal liver cancer lesion edges and the ablation zone edges. The minimum distance between the two is defined as the minimum ablation boundary. The plug-in can also automatically measure the 3D volume that does not reach the safe ablation distance.

The Dice similarity coefficient (Dice) is used to evaluate the performance of the segmentation model; the closer the Dice value is to 1, the better the segmentation effect is. The formula is as follows: given two binary segmentation maps RS and PS, which represent the label and segmentation results, respectively.

(1) $$\begin{array}{c} \text{DSC}=\frac{2\cdot \left|\text{RS}\cup \text{PS}\right|}{\left|\text{RS}\right|\cap \left|\text{PS}\right|}. \end{array}$$

In addition, the Fl score was used to assess the segmentation accuracy of liver tumor and ablation zone with the following equation: where TP is truly positive, FN is false negative and FP is a false positive.

(2) $$\begin{array}{c} \text{Sensitivity}=\frac{\text{TP}}{{\text{TP}}^{2}‐\text{F}{\text{N}}^{2}}. \end{array}$$

The *k*-nearest neighbor algorithm idea is very simple. Firstly, the observation objects in the training set are projected into the high-dimensional space based on their variable values, and each observation object is a point in the high-dimensional space. The more similar the variable properties between the observation objects, the closer the spatial distance of these points will be. Thus, similar observation objects exhibit a certain spatial aggregation in the high-dimensional space. In this study, when applying the model to the test set, each observation object in the test set is projected onto a high-dimensional spatial graph composed of the training set based on its variable information. The *k* points closest to each observation in the test set are selected, and if there are more liver cancer patients in the *k* points, the object is judged as liver cancer, and if there are more non-hepatocellular cancer patients, the object is judged as non-hepatocellular cancer, as shown in Figure 1.

His classification idea fits well with the clinician's diagnostic thinking and can construct concise and easy-to-understand rules. The shape of a decision tree resembles an inverted tree, which consists of a root node at the top of the decision tree, with edges emanating downward connecting inner nodes, and a leaf node at the bottom of the decision tree. The decision tree algorithm is a recursive division process. For the nodes, the decision tree calculates the information gain of each variable, and the information gain of different variables varies so that the “impurity” of the child nodes decreases differently according to their division [22]. The variable that causes the fastest decrease in “impurity” is the variable that builds the branch. For each branch, the above process is repeated to build new branches, which is the process of decision tree generation.

BP artificial neural network can continuously adjust the weight value of variable information transfer and Kan value of activation function in the whole network through error backpropagation, and this algorithm can make BP artificial neural network fit any form of continuity function. Therefore, BP artificial neural network has powerful nonlinear mapping ability and can process and mine the internal structure of complex data, which has good performance in medical image processing and clinical auxiliary diagnosis. Attention mechanism is a special structure that people embed in machine learning models to automatically learn and calculate the contribution of input data to output data. Attention mechanism is a data processing method in machine learning, which is widely used in various types of machine learning tasks such as natural language processing (NLP), image processing (CV), and speech recognition. According to the difference in the application of the attention mechanism to the domain, that is, the way and location of the attention weights, the attention mechanism is divided into three types: spatial domain, channel domain, and mixed domain.

## 4. Results Analysis

### 4.1. Experimental Results

To investigate the role of Mcl-1 in JQ1-triggered apoptosis in HCC cells, we first used two different siRNAs targeting different Mcl-1 gene sequences to knock down the expression level of Mcl-1 in the HCCLM3 cell line. Our results further revealed treatment of siCTL-transfected cells with 0.5uM JQ1 and western blotting results revealed that JQ1 induced caspase-3 activation and PARP cleavage, but the treatment of HCCLM3 cells with Mcl-1 knockdown at the same concentration of JQ1 resulted in almost complete cleavage of full-length PARP, while it only minimally reduced the level of full-length PARP in control cells.

These results suggest that JQ1 activates a stronger apoptotic signal when Mcl-1 is inhibited in HCC cells. In addition, flow cytometry combined with AnnexinV and PI double staining was used to detect apoptosis in HCCLM3 cells, and the apoptosis rates of transfected siMcl-1 (a) and siMcl-1 (b) cells were (64.7 ± 5.2) % and (70.7 earth 5.5) %, respectively, both of which were significantly higher than those of control cells (26.7 s-1.2) %. These results suggest that inhibition of Mcl-1 in this relatively sensitive HCCLM3 cell line further enhanced JQ1-mediated apoptosis in HCC cells, as shown in Figure 2.

When cell confocal fluorescence microscopy experiments were required, cells were grown and cultured using 35 mm laser confocal dishes. 35 mm laser confocal dishes have a bottom area equivalent to the size of a single well of a 6-well plate, with the special feature of a circular coverslip embedded in the bottom of the confocal dish for laser tool set microscopy, reducing a series of steps during the cell crawling operation and facilitating the experimental process. When using the laser confocal dish to grow cells, a pre-equilibration operation is required before adding cells, i.e., adding 1 mL of culture medium to the glass-bottom dish and then placing it in the incubator for 15 min, followed by the operation of adding cells and culture medium. The density of cell growing was 10,000 cells, and the next experimental operation such as drug addiction could be carried out in about 12 h. The cell growing density could be adjusted appropriately according to the interval of the next operation, as shown in Figure 3.

To further identify whether the changes in ATG4B acetylation level are related to ATG4B-mediated changes in autophagy function, we performed immunoprecipitation using anti-acetylation-specific antibodies to detect the changes in ATG4B acetylation after sorafenib treatment. The level of LC3-II was significantly increased after treatment with sorafenib, while the protein level of ATG4B did not change significantly after treatment with sorafenib, but the level of acetylation of ATG4B was significantly decreased, suggesting that the decrease in the level of acetylation of ATG4B may lead to LC3, the reason for the enhanced level of -II. Decision tree is a very classic algorithm, a non-parametric supervised learning method that can solve classification and regression problems. A decision tree makes decisions based on a tree-like structure. A decision tree contains a root node, several branches, several internal nodes, and several leaf nodes. The root node represents the complete set of samples, the branches represent the output of a judgment result, and the internal nodes represent an attribute. The judgment of the leaf node represents a classification result.

### 4.2. Preliminary Diagnostic Results

The continuous variables were standardized, the correlation matrix between the variables was sought, the independent variables were diagnosed for covariance, and the variables with strong correlation were adjusted for variance inflation factor no greater than 10 by combining them into new variables or directly deleting one of them to achieve the purpose of controlling multicollinearity. The variables with statistically significant differences in the single-factor analysis were subjected to multi-factor analysis, the equations were constructed using a generalized linear model, and the Sigmoid function was selected for the linkage function. The forward likelihood ratio method was used to screen the variables. The model was validated in the test set. The diagnostic efficacy of the model was evaluated by the area under the ROC curve, sensitivity, specificity, and accuracy.

In this study, the training and test sets were obtained by one stratified random sampling. Due to sampling error, the training and test sets may have specific distributional characteristics that may lead to the particularly good performance of some models or particularly poor performance of others. In this study, the error rate is chosen to describe the diagnostic effectiveness of the model. For each fold of cross-validation, one error rate of the model is obtained in both the training set and the test set; 10-fold cross-validation is then able to obtain 10 error rates in each of the training and test sets. The mean and standard deviation of the 10 error rates is more robust to the diagnostic performance of the model. An elusive goal of pain research is the identification of objective markers of chronic pain states. Ideally, this marker is more pronounced in chronic pain patients and can be quantitatively tracked according to the severity of clinical pain perception. In traumatic pain, such as fibromyalgia (FM), altered central nervous system function contributes to the perception of pain without surrounding tissue damage or inflammation. Resting-state fMRI can provide insight into the inner dynamics of the brain by measuring functional connectivity.

The BP neural network model performed best in the training set, with a mean and standard deviation of 10-fold cross-validation of 10.50s for the percent error rate, which was better than 13.34 s for the decision tree, 13.52 s for the weighted *k*-nearest neighbor, and 16.28 s for the logistic regression, all with statistically significant differences. The standard deviation of the error rate of BP artificial neural network and logistic regression is smaller, so the fluctuation of these two models in the training set is also smaller, as shown in Figure 4.

The early diagnosis model of hepatocellular carcinoma constructed by using the existing routine serological examination indexes is the focus of this study. The model can not only assist clinicians in the early diagnosis of liver cancer but also has some early liver cancer screening functions for the general consultation population. To fully explore the relationship between each index and liver cancer, four machine learning classification methods: logistic regression, weighted *k*-nearest neighbor, decision tree, and BP artificial neural network were used to construct the liver cancer model in this study.

The results showed that the BP neural network model in the training set had the highest diagnostic efficacy for liver cancer, outperforming decision trees, weighted *k*-nearest neighbors, and logistic regression. The standard deviation of the error rates of BP artificial neural network and logistic regression models were smaller, so the error rates of these two models also fluctuated less in the training set.

The results in the training set suggest that the BP artificial neural network model may maximize the internal structure and correlation information of the data in the training set, while the logistic regression model extracts the main information but ignores some details, so the performance of both models is relatively stable. The weighted *k*-neighborhood only uses the label information of the nearest *k* samples in the determination and cannot use all the information of the training set, which may be the main reason for the unstable performance of the model. The essence of the decision tree is the division of space, so it relies heavily on the spatial distribution of the samples in the training set, and different spatial distributions may lead to large differences in the diagnostic performance of the decision tree model, as shown in Figure 5.

The BP neural network model had the highest diagnostic efficacy for liver cancer in the test set, outperforming the decision tree, weighted *k*-nearest neighbor, and logistic regression models. The decision tree outperformed the weighted *k*-nearest neighbor and logistic regression models. The weighted *k*-nearest neighbor and logistic regression models had comparable diagnostic efficacy. The standard deviation of the error rates of all four models in the test set was relatively large, and therefore, the error rates of all four models fluctuated more in the test set. The diagnostic performance of the diagnostic models constructed by BP neural network, weighted *k*-nearest neighbor, and decision tree was better in the training set than in the test set. The diagnostic performance of the logistic regression model did not differ between the training and test sets.

In this study, potential TAAbs for liver cancer were screened based on a custom-made high-throughput proteomic microarray and further screened using KEGG cancer pathway analysis from the String database and positive rates in the liver cancer and control groups. The enzyme-linked immunosorbent assay (ELISA) was used to detect and validate the diagnostic value of anti-TAAs autoantibodies for liver cancer for the screened TAAbs, and the levels of anti-TAAs autoantibodies in liver cancer patients, cirrhotic patients, hepatitis B patients, and healthy controls were examined to assess the possible time points of tabs. Multiple diagnostic models for liver cancer were constructed using data mining techniques to explore the value of combined TAAbs detection in liver cancer screening and diagnosis, from which the optimal model was selected to evaluate the diagnostic value of each tab and the optimal model for different clinical subgroups of liver cancer.

## 5. Conclusion

The apoptosis of cells was detected by flow cytometry, i.e., the apoptosis rate was higher in the si-SIRT group than in the si-Ctrl group, so it can be indicated that inhibition of the SIRT1 gene can promote apoptosis of hepatocellular carcinoma cells, and this conclusion was verified by protein immunoblotting with increased levels of apoptosis-related caspase-3 and PARP. CD44 molecules overexpressed on the tumor cell surface were used as targets. The obtained nanoparticles possess strong emission fluorescence properties and a high magnetization rate and have a good biosafety profile. Under white light irradiation, the nanoparticles can generate large amounts of reactive oxygen species for photodynamic therapy. Decision trees are essentially a partitioning of a high-dimensional space, and the decision tree model fitting process is independent of the sample size and the type of variables. The decision tree also has a certain ability to analyze the causes, and the variables used to classify the nodes have a strong correlation with liver cancer. The number of studies with sensitivity and specificity data for AFU + AFP combined diagnosis of HCC is too small to allow heterogeneous meta-regression analysis, which affects the credibility. Publication bias exists between studies, and the high heterogeneity of the diagnostic indicators studied and the inability to eliminate heterogeneity lead to a decrease in the reliability of the results.

## Figures and Tables

**Figure 1:** Principle of decision tree.

**Figure 2:** Average percentage of apoptotic cells in the experiments.

**Figure 3:** Induction of protective autophagy in hepatocellular carcinoma cells.

**Figure 4:** Comparison of error rates in the training set and test set for the four classification models.

**Figure 5:** ROC curves of logistic regression model for early and late-stage liver cancer diagnosis.

**Table 1:** Basic characteristics of the study subjects.

Features	Small sample				Big sample			
	Hepatic carcinoma	Control group	*Z*	*P*	Hepatic carcinoma	Control group	*Z*	*P*
N	62	63	2	4	120	133	2	3
Man	57.3	64.2			37.8	56.3		
Woman	82.1	80			83.2	79.2		
Age	25	25			25	25		
BCLC A	20				27			
BCLC B	24				24			
BCLC C	26				21			
BCLC D	11				15			
AFP(+)	47.8				72.1			
AFP(-)	26.5				40.4			
Size≤5 cm	27.0				55.1			
Size>5 cm	64.4				62.3			

**Table 2:** Relevant experimental drugs and equipment.

No.	Reagent	Quantity	Production
1	SIRT1-siRNA	2	Hyclone
2	RiboFECT™ CP reagent	4	Hyclone
3	RiboFECT™ CP buffer	2	Hyclone
4	DMEM	20	Hyclone
5	0.35% High glucose medium	5	Hyclone
6	24 pores	6	Corning
7	Caspase-3	4	CST
8	RAPR	3	Abcom
9	*β*-Actin	5	Proteintech
10	1.5 mL LEP	9	Biosharp
11	Annexin V-FITC	11	BD
12	SDS-PEAG(5×)	12	Biosharp

**Table 3:** Structural parameters of the two-dimensional RA-Unit network for liver segmentation.

Encoder	Output size	Decoder	Output size
Input	128 × 128 × 64	Attention block 1	256 × 128 × 1
Residual block 1	128 × 128 × 128	Residual block 6	256 × 128 × 1
Pooling	32 × 1 × 512	Convolution	256 × 64 × 32
Residual block 2	128 × 128 × 1	Attention block 2	512 × 512 × 1
Pooling	128 × 128 × 1	Residual block 7	512 × 512 × 1
Residual block 3	128 × 32 × 1	Convolution	256 × 64 × 32
Pooling	128 × 128 × 1	Attention block 3	256 × 64 × 32
Residual block 4	64 × 64 × 64	Residual block 8	256 × 128 × 1
Pooling	32 × 1 × 512	Convolution	64 × 64 × 64
Residual block 5	512 × 512 × 1	Attention block 4	32 × 1 × 512
Convolution	256 × 64 × 32	Residual block 9	32 × 1 × 512
Pooling	128 × 128 × 1	Convolution	1 × 64 × 64

## Data Availability

The data used to support the findings of this study are available from the corresponding author upon request.
